The article "How the Malaria Vector Anopheles gambiae Adapts to the Use of Insecticide-Treated Nets by African Populations" was retracted in 2016. Reasons: fabricated or falsified data; concerns about the data; concerns about the results or conclusions.

# How the Malaria Vector *Anopheles gambiae* Adapts to the Use of Insecticide-Treated Nets by African Populations

**DOI:** 10.1371/journal.pone.0097700

**Published:** 2014-06-03

**Authors:** Mamadou Ousmane Ndiath, Catherine Mazenot, Cheikh Sokhna, Jean-François Trape

**Affiliations:** 1 G4-Group, Institut Pasteur International Network, Entomology Unit, Institut Pasteur of Bangui, Bangui, Central African Republic; 2 Laboratoire de Paludologie et de Zoologie Médicale, Institut de Recherche pour le Développement, Campus International UCAD- IRD, Hann, Dakar, Sénégal; 3 Unité de Recherche sur les Maladies Infectieuses et Tropicales Emergentes, IRD198, UM63, CNRS7278, INSERMU1095, Aix-Marseille Université, Campus UCAD-IRD, BP 1386, Dakar, Sénégal; University of Queensland & CSIRO Ecosystem Sciences, Australia

## Abstract

**Background:**

Insecticide treated bed nets have been recommended and proven efficient as a measure to protect African populations from malaria mosquito vector *Anopheles* spp. This study evaluates the consequences of bed nets use on vectors resistance to insecticides, their feeding behavior and malaria transmission in Dielmo village, Senegal, were LLINs were offered to all villagers in July 2008.

**Methods:**

Adult mosquitoes were collected monthly from January 2006 to December 2011 by human landing catches (HLC) and by pyrethroid spray catches (PCS). A randomly selected sub-sample of 15–20% of *An. gambiae s.l.* collected each month was used to investigate the molecular forms of the *An. gambiae* complex, kdr mutations, and *Plasmodium falciparum* circumsporozoite (CSP) rate. Malaria prevalence and gametocytaemia in Dielmo villagers were measured quarterly.

**Results:**

Insecticide susceptible mosquitoes (wild kdr genotype) presented a reduced lifespan after LLINs implementation but they rapidly adapted their feeding behavior, becoming more exophageous and zoophilic, and biting earlier during the night. In the meantime, insecticide-resistant specimens (kdr L1014F genotype) increased in frequency in the population, with an unchanged lifespan and feeding behaviour. *P. falciparum* prevalence and gametocyte rate in villagers decreased dramatically after LLINs deployment. Malaria infection rate tended to zero in susceptible mosquitoes whereas the infection rate increased markedly in the kdr homozygote mosquitoes.

**Conclusion:**

Dramatic changes in vector populations and their behavior occurred after the deployment of LLINs due to the extraordinary adaptative skills of *An. gambiae s. l.* mosquitoes. However, despite the increasing proportion of insecticide resistant mosquitoes and their almost exclusive responsibility in malaria transmission, the *P. falciparum* gametocyte reservoir continued to decrease three years after the deployment of LLINs.

## Introduction

The preventive measures against malaria recommended by WHO include anti-vectorial procedures such as indoor residual spraying (IRS), use of long-lasting insecticide-treated bed nets (LLINs) and destruction of larvae breeding sites [1]. The presence of insecticide treated materials inside the habitation has consequences on the vector populations, reducing density, survival, contact with humans and feeding frequency [2], [3], [4]. As a result, in areas where LLINs have been used, malaria transmission, prevalence, morbidity and mortality have decreased significantly [2], [5], [6], [7], [8], [9].

*Anopheles* vectors are known to display remarkable adaptation skills that enable their survival in widely varying environmental conditions [10]. Although the use of insecticide reduces mosquito density, it has led to the selection of resistant strains [11], [12], [13], [14]. Multiple mechanisms of resistance to insecticides have been observed in anopheline populations, including target site mutation (kdr) and increased metabolic detoxification [15]. Behavioural modifications have also been reported in mosquitoes exposed to insecticide, such as a shift from endophilic to exophilic behaviour and changes in time of feeding [16], [17], [18], [19]. LLINs remain an effective tool to reduce the burden of malaria, but the long term effects of insecticide on vector populations and malaria transmission remain to be evaluated.

Indeed, the long term efficacy of LLINs in reducing malaria morbidity has recently been questioned in Western Africa, both in a rural area of Senegal, with evidence of a rebound in malaria morbidity, coinciding with the emergence notably the kdr mutation [20], [21] and in Benin were universal coverage with LLINs and/or IRS have shown no benefit on morbidity in comparison to target LLINs use [22]. In the present study, we examined the changes in the principal malaria mosquito vectors following implementation of a universal coverage with LLINs (Permanet 2) in July 2008. Vector density, composition, malaria transmission and behavioural characteristics were studied in the light of emerging insecticide-resistant mosquitoes, 31 months before and 41 months after the generalized use of LLINs and related to changes in malaria epidemiology.

## Materials and Methods

### Mosquito sampling

This study is part of the Dielmo Project that has been described in details elsewhere [23]. Briefly, the village of Dielmo (13°43′N, 16°24′W) is located 280 km southeast of Dakar and about 15 km north of the Gambian border in an area of Sudan-type savannah. About 500 inhabitants are living in the village. Rainfall occurs during a four-month period, from mid-June to mid-October. Dielmo is situated on the marshy bank of a small permanent stream, with anopheles breeding sites present all year round. During the second week of July 2008, all villagers were offered long-lasting deltamethrin-treated nets (LLINs) (Permanet 2.0). Household visits were conducted quarterly to confirm ownership and to monitor their use and condition. During these household visits, ownership of bednets in the study population after the implementation of LLINs was respectively 97.7% in 2008 and 95.6 in 2011. LLINs of all villagers were renewed in July 2011 after we documented a rebound in malaria morbidity. There were no LLINs in Dielmo before July 2008. A detail description of the study area and the history of different malaria treatments were given previously [20], [23].

Adult mosquitoes were collected monthly from January 2006 to December 2011. Night human landing catches (HLC) were conducted two or three nights each month, between 7:00 PM and 7:00 AM, in two indoor and two outdoor sites. In each site, two trained collectors (adult male volunteers) worked alternatively for one hour and rested for one hour. Pyrethroid spray catches (PCS) were performed at 7:00 AM by spraying Deltamethrin (Yotox) for 30–45 seconds in a room. After 10 minutes, dead and immobilized mosquitoes were collected. Anopheline identification was performed following morphologic identification keys [24]. Sampling sites were the same throughout the whole study time. Except LLINs and PSC, no other insecticide was used in the village.

### Laboratory analyses

Infection rates were determined in all anophelines by performing ELISA with monoclonal antibodies against *Plasmodium falciparum* Circumsporozoite Protein (CSP) on the crushed head and thorax [25]. In a randomly selected sub-sample of 15–20% of *An. gambiae s.l.* collected each month, the identification of L1014F and L1014S kdr mutations was performed by PCR according to Martinez-Torres and al. and Ranson and al. [26], [27] and identified of sub-species and molecular forms by PCR RFLP [28] on the carcasses of dissected mosquitoes. Blood fed females captured by PSC had their blood meal squashed on Whatman No. 1 filter papers and tested by ELISA to identify whether blood was of human or animal origin [29].

### Epidemiologic data

*Plasmodium falciparum* gametocyte prevalence and density were measured quarterly from 2006 to 2011 in all residents of the village enrolled in the project. Blood was taken using a finger prick and we examined 200 oil-immersion fields (approximately 0.5 µl of blood) with a first reading in the field followed by laboratory confirmation.

### Data analysis

Rates were compared using Fisher exact and Pearson Chi^2^ tests, quantitative data by non parametric Mann-Whitney or Kruskal-Wallis tests. Multivariate analyses were performed using logistic models (Likehood ratio and Wald Chi^2^ are reported). Statistical analyses were performed using Stata 10.1 software. A P value of 0.05 or less was considered as significant.

### Ethics approval

The Dielmo project was initially approved by the Ministry of Health of Senegal and the assembled village population. Approval was then renewed on a yearly basis. Audits were regularly conducted by the National Ethics Committee of Senegal and ad-hoc committees of the Ministry of Health, the Pasteur Institute and the Institut de Recherche pour le Développement. Written informed consents were obtained individually from all participants in our study or the parents of children younger than 15 years.

## Results

### Species density

From January 2006 to December 2011, 14,292 *Anopheles* specimens were sampled, by HLC during 744 man night captures; among them 8,855 (62.0%) were *Anopheles gambiae sensu lato* and 5,190 (36.3%) *Anopheles funestus* (Table 1 in File SI).

The human biting rate (HBR) of *An. gambiae s.l.* remained stable from 2006 to 2011 and was always highly seasonal (Figure A in File SI). The implementation of LLINs had little influence on HBR (11.8 bites/man/night before *vs*. 12.0 after). The Entomological Inoculation Rate (EIR) of *An. gambiae*, decreased temporarily in 2009, i.e. the year after the implementation of LLINs (0.14 infected bites/man/night *vs*. 0.22 to 0.34 between 2006 and 2008), but increased again in 2010 and 2011 (0.24 and 0.21 respectively). When calculated globally, EIR only slightly decreased during the period after the implementation of LLINs (0.18 infected bite/man/night vs. 0.33 before).

A subsample of 1,494 *An. gambiae s.l.* was used for taxa identification. Among them 24.6% were classified as *An. arabiensis*, 25.5% *An. coluzzii* (previously molecular form M), 49.7% *An. gambiae* molecular form S, and only 0.2% hybrids (*An. coluzzii* and molecular form S) (Table 2 in File SI). The proportion of *An. gambiae* molecular form S decreased in 2008 and 2009 (just after the implementation of LLINs) and increased again in 2010 and 2011 (Pearson Chi^2^<0.001). By contrast, the proportion of *An. coluzzii* and *An. arabiensis* increased in 2008 and 2009 (Pearson Chi^2^<0.001, Table 2 in File SI).

*An. funestus* was present all year round before LLINs; they almost disappeared after July 2008 only to reappear in September 2010 (SI Figure A in File SI). HBR dropped from 17.2 bites/man/night during the period before LLINs to 1.2 after. The EIR of *An. funestus* was 1.2 infected bites/man/night before LLINs, but zero from August 2010 to the end of 2011.

### Kdr genotypes

No *Anopheles* specimen with L1014S kdr mutation was identified in the study. Specimens with L1014F (hereafter referred to as kdr R) allele were detected at a low and constant rate from 2006 to 2008 (Table 2 in File SI). A significant increase in R allelic frequency was observed in 2009 (9.72% *vs*. 2.92% in 2006–2008, Pearson Chi^2^ p<0.001), with a dramatic rise in 2010 (23.16%) and 2011 (30.86%, Pearson Chi^2^ p<0.001 in both cases). The relative frequency of RR and RS genotype was higher in *An. gambiae* molecular form S than in *An. coluzzii* or in *An. arabiensis*.

### Feeding time

Hourly aggressiveness of *An. gambiae s.l.* analyzed by kdr genotype group, after the implementation of LLINs, showed a shift of aggressiveness to earlier hours (09:00 PM to 01:00 AM) in the SS group (Fig. 1 panel A). This resulted in an earlier median feeding time in the SS kdr group after LLINs vs. before (Man-Whitney test p<0.0001, Fig. 1 panel B). No significant change was observed in the RS genotype group. During the period after LLINs, SS genotype specimens had a significantly earlier median feeding time than RS and RR specimens (Kruskal-Wallis test p<0.0001).

**Figure 1:** An. gambiae feeding time measured in 1494 An. gambiae s.l. mosquitoes sampled from 2006 to 2011, according to their kdr genotype (SS: wilde type, yellow lines and boxes, RS: L1014 F heterozygote, orange lines and boxes, RR: L1014F homozygote, red lines and box). Panel A represents hourly aggressiveness in specimens sampled each hour after the implementation of LLINs as a percentage of the number of specimen sampled during the night. Panel B boxes are 25th to 75th percentiles with median hour, lines are 1.5 interquartile and dots outside values, for specimens sampled from Jan 2006 to Jul 2008 (Before LLINs) and between August 2009 and Dec 2011 (After LLINs). Changes in median hour of aggressiveness observed in the SS specimen group after the implementation of LLINs (Mann-Whitney test p<0.0001) but not in RS specimens. Earlier aggressiveness detected in SS group in comparison to RS and RR after LLINs (Kurskal-Wallis test p<0.0001).

### Parity rate

Parity rate in the *Anopheles* population significantly changed over time during the study (Fig. 2, panel A): it decreased in 2008 and 2009 in comparison to 2006 (Fisher p<0.001) and increased in 2010 to a value that was not significantly different from 2006 and again in 2011(p<0.005 vs. 2006 and p<0.001 vs. 2010). The same changes were observed in all three taxa groups (Fig. 2 panel B). From 2006 to 2008, no significant difference was observed in parity rate among kdr groups. From 2009 to 2011, parity rate was significantly lower in the SS group than in the RS and RR groups (Fisher p = 0.02, 0.01 and 0.03 in 2009, 2010 and 2011 respectively).

**Figure 2:** Parity rate (% and 95% confidence interval) measured in 1494 *An. gambiae s.l.* mosquitoes sampled from 2006 to 2011, according to their kdr genotype (SS: wilde type yellow box, RS: L1014 F heterozygote orange box, RR: L1014F homozygote red box, Panel A) and taxa (*An. arabiensis*, green boxes, *A. coluzzi*, light blue boxes, and *An. gambiae* form S, darck blue boxes, Panel B). Rates in the total *Anopheles gambiae s.l.* population are given in brakets. Data in the table represent Odd ratio (OR) obtained with a logistic model of parity with following factors: KDR genotype, taxa and year. Likehood ratio Chi^2^ = 244.72, p<0.001.

In a logistic model adjusted on taxa and year, KDR genotype was significantly associated with parity with both RS and RR groups being more pareous than SS group. When adjusted on KDR and year, taxa group were not significantly associated with parity (Chi^2^ = 2.14, p = 0.54). When adjusted on KDR groups and taxa, parity was significantly associated with trial year with a reduced parity in 2008, 2009 and 2010.

### Endophagic behaviour

Endophageous rate significantly changed over time in the *Anopheles* population (Pearson Chi^2^ p<0.001, Fig. 3 panel A). Endophageous rate did not significantly vary in both RR and RS genotype groups (Pearson Chi^2^ = 0.5 and 0.6 respectively), it significantly dropped in 2010 and 2011 in comparison to 2009 in the SS group (Pearson Chi^2^<0.001 for both years). SS specimens were less endophagic than other genotypes even before the implementation of LLINs but this difference was much more dramatic in 2010 and 2011. When studied among taxa, exophagic behaviour significantly changed. Especially, endophageous rate of *An. arabiensis* decreased from 2008 to 2011 and endophageous rate of *An. gambiae* S decreased in 2008 only (Fig. 3 panel B).

**Figure 3:** Endophageous rate (% and 95% confidence interval) measured in 1494 *An. gambiae s.l.* mosquitoes sampled from 2006 to 2011, according to their kdr genotype (SS: wilde type yellow box, RS: L1014 F heterozygote orange box, RR: L1014F homozygote red box, Panel A) and taxa (*An. arabiensis*, green boxes, *An. coluzzii*, light blue boxes, and *An. gambiae* molecular form S, darck blue boxes, Panel B). Rates in the total *Anopheles gambiae s.l.* population are given in brakets. Data in the table represent Odd ratio (OR) obtained with a logistic model of parity with following factors: KDR genotype, taxa and year. Likehood ratio Chi^2^ = 330.68, p<0.001.

In a logistic model adjusted on taxa and year of study, the KDR group is significantly associated with the endophageous rate, with both RS and RR groups having an increased endophagy in comparison to SS KDR group. Taxa groups were also significantly associated with the endophageous rate when adjusted on KDR and year with both *An. coluzzii* and *An. gambiae* S form being more endophageous than *An. arabiensis*. The year of study was also associated with the endophageous rate when adjusted on KDR and taxa groups, with specimens sampled in 2007 and 2009 being more endophageous than in 2006, and in 2011 being less endophageous than those sampled in 2006.

### Human Blood Index

Blood meal origin was analyzed on *An. gambiae* mosquitoes specimens (n = 735) sampled by PSC from 2006 to 2011 (SI Table 3). HBI was constant and not different in the two kdr groups in 2006 and 2007, it significantly dropped from 2008 to 2011 in the kdr SS group in comparison to RS and RR groups and baseline value (Pearson chi^2^ p<0.01, Fig. 4 panel A). From 2009 to 2011, kdr RR specimens always fed exclusively on humans. Anthropophilic rate in SS kdr group was reduced after the implementation of LLINs (40.5% vs 79.3% before, Pearson chi^2^ p<0.001) but not in RS group (77.2% vs 100%). Antropophilic rate reduction from 2009 was observed in all taxa and was maximal in *An. arabiensis* (Fig 4 panel B).

**Figure 4:** Human blood index (HBI) (% and 95% confidence interval) measured in 735 *An. gambiae s.l.* mosquitoes sampled from 2006 to 2011, according to their kdr genotype (SS: wilde type yellow box, RS: L1014 F heterozygote orange box, RR: L1014F homozygote red box, Panel A) and taxa (*An. arabiensis*, green boxes, *An. coluzzii*, light blue boxes, and *An. gambiae* molecular form S, darck blue boxes, Panel B). Rates in the total *Anopheles gambiae s.l.* population are given in brakets. Data in the table represent Odd ratio (OR) obtained with a logistic model of parity with following factors: KDR genotype, taxa and year. Likehood ratio Chi^2^ = 113.49, p<0.001.

In a logistic model adjusted on taxa and year, KDR genotype was significantly associated with HBI with RS group feeding more on human than SS group (Wald Chi^2^ 19.52, p>0.0001). 100% (18/18) of RR specimens fed on human. When adjusted on KDR and year, taxa group were significantly associated with HBI with both *An. gambiae* S and *An. coluzzii* feeding more on human than *An. arabiensis* (Wald Chi^2^ = 22.71, p<0.0001). When adjusted on KDR groups and taxa, HBI was significantly associated with trial year with a reduced HBI from 2008 to 2011 (Wald Chi^2^ 71.65, p>0.0001).

### Infection rates

In the total sampled *An. gambiae s.l.* population (n = 8,855), the CSP rate did not change during the 2006–2008 period, but significantly dropped in 2009 (0.79% vs. 2.49% during the 2006–2008 period, Pearson Chi^2^ p<0.001) (Fig 5). CSP rate significantly increased in 2010 (1.87% p = 0.002 vs. 2009) and again in 2011 (3.09% p = 0.04 vs. 2010 value) to reach values that were not significantly different from those observed during the 2006–2008 period.

**Figure 5:** Circumsporozoite Protein (CSP) rate (% and 95% confidence interval) measured in 1494 *An. gambiae s.l.* mosquitoes sampled from 2006 to 2011, according to their kdr genotype (SS: wilde type yellow box, RS: L1014 F heterozygote orange box, RR: L1014F homozygote red box). CSP rate in the total sampled population (n = 8,855) is given in brackets at the bottom of the figure. Data in the table represent Odd ratio (OR) obtained with a logistic model of parity with following factors: KDR genotype, taxa and year. Likehood ratio Chi^2^ = 69.06, p<0.001.

When measured in the kdr genotyped sub-sample, infection rate was low and similar in both SS and RS groups from 2006 to 2008 (Fig. 5). From 2009 to 2011, infection rate in RR genotype group was spectacularly high and globally after LLINs it reached 25.5%. By contrast, infection rate in RS genotype group decreased after 2008. It reached a global value of 1.2% after LLINs vs. 4.6% before. Infection rate in SS group was 3.8% before LLINs, no single infected SS mosquitoes were found after their implementation.

In a logistic model adjusted on taxa and year, the risk of infection with *P. falciparum* was significantly associated with KDR genotype (Wald test Chi^2^ = 42.95 p<0.001) with RR specimen having an increased risk in comparison to SS genotype. Taxa groups were not significantly linked to infection when adjusted on KDR genotype and year (Wald test Chi^2^ = 0.51, p = 0.78). The risk of being infected, adjusted on KDR and taxa groups significantly decreased in 2009, 2010 and 2011 (i.e. after the implementation of LLINs) in comparison to 2006 (Wald test Chi^2^ = 36.76 p<0.001).

### Gametocytemia

Between 2006 and 2011, the prevalence of gametocyte carriers in the general population gradually decreased from 7.05% to 1.07% (Pearson Chi^2^ = 105.38, p<0.001, Table 4 in File SI). Although the mean gametocytemia in positive patients did not significantly change (Kruskal Wallis p = 0.75, Table 4 in File SI). The proportion of *P. falciparum* infections with gametocytes increased from 22.6% in 2006 to 46.4% in 2010 and 42.1% in 2011 (Pearson Chi2 = 13.6, p<0.02, Table 4 in File SI).

## Discussion

This study demonstrates the exceptional adaptability of *Anopheles* to the presence of insecticide. A series of adaptative processes were observed in the *An. gambiae s.l*. population after mass deployment of LLINs inside houses. Firstly, mosquitoes that remained susceptible to insecticide had a marked decreased lifespan after LLINs implementation. In the following years, they tended to adapt by shifting to outdoors host seeking, by biting earlier and increasing feeding on animals. Secondly, insecticide-treated nets quickly selected resistant mosquitoes with long lifespan and unchanged feeding behaviour. This change in species composition following LLINs implementation has been previously noted for *An. arabiensis* [30], [31] and likely reflects its known opportunistic host choice, feeding on both humans and animals. Although *An*. *funestus* in Dielmo fluctuated markedly from 1990 to 2007 [23], [32], the implementation of LLINs coincided with the total suppression of the role of *An*. *funestus* in malaria transmission. Unlike *An. gambiae*, *An. funestus* in Dielmo did not present kdr mutation but rather behavioural changes on biting hours with peaks of maximum aggressiveness in broad daylight between 07:00 and 11:00 AM [19].

The selection of resistant specimens by the use of insecticide-treated materials has already been widely reported [11], [14]. This study demonstrates that the R allelic frequency rose shortly after the implementation of LLINs and continued to increase three years later. The presence of the kdr mutation has been shown to be associated with a reduced susceptibility to pyrethroids and DDT [21] although other resistance mechanisms should also be taken into account.

On the other hand, changes in feeding time following the use of LLINs have already been observed in other studies, reporting either a shift to early feeding, just after sunset or to morning feeding just before sunrise [16], [18], [19]. Our study demonstrates that changes in aggressiveness exclusively involved the SS genotype sub-group that is potentially the most susceptible to insecticide. Equally, as previously demonstrated in other studies [8], [31], the presence of insecticide treated materials inside houses decreased mosquito lifespan in the years following their implementation. Our study shows that this reduction was particularly important in kdr SS specimens that were the most susceptible to insecticide. However, parity rates remained constant in the RR kdr genotype, demonstrating the lack of insecticide killing effect in this group. In the past few years, even kdr SS specimens have a high parity rate. This may be explained by the selection of *An. gambiae* specimens having acquired other mechanism of resistance, different from kdr mutation [21]. The longer lifespan in RR specimens may explain the high CSP rate observed in this group. This would suggest that adaptative mechanisms to insecticide have promoted survival to the detriment of reproduction, leading to few but highly infectious females.

Shift from endophagic to more exophagic host seeking behaviour in *An. gambiae s.l.* has been reported in various studies after the implementation of insecticide-treated materials inside houses [16], [17]. In the present work, the mass use of LLINs have been associated with increased exophagic behaviour, especially in species with opportunistic feeding behaviour such as *An. arabiensis* and in the most susceptible to insecticide such as SS mosquitoes. All these data demonstrate that insecticide susceptible mosquitoes adapted to the presence of LLINs inside houses by feeding more on animals. These changes occur in *An. arabiensis* that is known to have an opportunistic feeding behaviour [33] but also in *An. gambiae s.s.* which is remarkable and demonstrates its outstanding adaptiveness.

Although the decreased infection rate in vectors after implementation of LLINs has already been reported [31], [34], this study is, to our knowledge, the first to identify subgroups inside *An*. *gambiae* complex that displays opposite behaviour regarding infection. Indeed, since the implementation of LLINs, infection rates dropped in SS and RS groups but significantly increased in the RR group that is now almost the only *P. falciparum* vector and plays a key role in the rebound of malaria morbidity observed in this population [20].

Whereas malaria-related morbidity dropped in the year following the implementation of LLINs [20], a reservoir of gametocyte carriers was still available for mosquitoes' infection. Furthermore, in 2010 and 2011, most all *P. falciparum* infections were associated with clinical malaria attacks, whose incidence density in older children and adults (but not in young children) returned to levels close to before the implementation of LLINs although very low levels of malaria prevalence persisted. Data analysis suggests that the choice of ACT used for first-line treatment and the universal deployment of LLINs were the most important factors governing the dramatic changes in anopheles populations and malaria morbidity. We hypothesize that these gametocytemia associated with clinical attacks may be more infectious to mosquitoes than those associated with asymptomatic infections. This could therefore explain maintenance of significant levels of transmission [35].

Despite the rapidly increasing insecticide resistant vector population and its almost exclusive responsibility in malaria transmission, the gametocyte reservoir continued to decrease three years after the deployment of LLINs. This support the view that it is important to pursue the use of LLINs in compliance with the WHO recommendations [1]. However, further research is urgently needed to face the problem of insecticide resistance that may rapidly compromise the recent successes of malaria control in tropical Africa.

## Supporting Information

File S1 **Supporting figure and tables.** SI Figure A Human Biting Rate (HBR, number of *Anopheles* sampled per man and per night, bars) and Entomological Inoculation Rate (EIR, number of infected *Anopheles* sampled per man and per night, dotted lines) in *A. funestus* (red) and *An. gambiae* (green) sampled each month from Jan 2006 to Dec 2011, before and after the implementation of long lasting insecticide treated nets (LLINs). SI Table 1. Number of specimens of each *Anopheles* species sampled during monthly human landing catches indoor and outdoor from 2006 to 2011. SI Table 2. Number of *An. gambiae* sampled and genotyped for (1) L1014F mutation (kdr) with heterozygote (RS), homozygote (RR), wild type (SS) and L1014F (R) allelic frequency (%), (2) *An. arabiensis, An. coluzzii* and *An. gambiae* S. SI Table 3. Number of *An. gambiae* collected 2006 to 2011 by pyrethrum spray catch (PSC) and genotyped for (1) L1014F mutation (kdr) with heterozygote (RS), homozygote (RR), wild type (SS) and the mean of human blood index (%), (2) *An. arabiensis, An. coluzzii* and *An. gambiae* S. SI Table 4. Number of *P. falciparum* gametocytes per 200 oil immersion fields in gametocyte positive slides (mean ± standard error of the mean), gametocyte prevalence (% and number of villagers with gametocytes/total villagers examined), and proportion of *P. falciparum* infections with gametocytes (% and number of villagers with gametocytes/number of villagers with *P. falciparum* infection). Dielmo, quarterly transversal surveys, 2006–2011.
(DOCX)
